# Lycopene Inhibits NF-kB-Mediated IL-8 Expression and Changes Redox and PPARγ Signalling in Cigarette Smoke–Stimulated Macrophages

**DOI:** 10.1371/journal.pone.0019652

**Published:** 2011-05-19

**Authors:** Rossella E. Simone, Marco Russo, Assunta Catalano, Giovanni Monego, Kati Froehlich, Volker Boehm, Paola Palozza

**Affiliations:** 1 Institute of General Pathology, Catholic University, Rome, Italy; 2 Institute of Nutrition, Friedrich-Schiller-Universität, Jena, Germany; 3 Institute of Anatomy, Catholic University School of Medicine, Rome, Italy; Istituto Dermopatico dell'Immacolata, Italy

## Abstract

Increasing evidence suggests that lycopene, the major carotenoid present in tomato, may be preventive against smoke-induced cell damage. However, the mechanisms of such a prevention are still unclear. The aim of this study was to investigate the role of lycopene on the production of the pro-inflammatory cytokine IL-8 induced by cigarette smoke and the possible mechanisms implicated. Therefore, human THP-1 macrophages were exposed to cigarette smoke extract (CSE), alone and following a 6-h pre-treatment with lycopene (0.5–2 µM). CSE enhanced IL-8 production in a time- and a dose-dependent manner. Lycopene pre-treatment resulted in a significant inhibition of CSE-induced IL-8 expression at both mRNA and protein levels. NF-kB controlled the transcription of IL-8 induced by CSE, since PDTC prevented such a production. Lycopene suppressed CSE-induced NF-kB DNA binding, NF-kB/p65 nuclear translocation and phosphorylation of IKKα and IkBα. Such an inhibition was accompanied by a decrease in CSE-induced ROS production and NOX-4 expression. Lycopene further inhibited CSE-induced phosphorylation of the redox-sensitive ERK1/2, JNK and p38 MAPKs. Moreover, the carotenoid increased PPARγ levels which, in turn, enhanced PTEN expression and decreased pAKT levels in CSE-exposed cells. Such effects were abolished by the PPARγ inhibitor GW9662. Taken together, our data indicate that lycopene prevented CSE-induced IL-8 production through a mechanism involving an inactivation of NF-kB. NF-kB inactivation was accompanied by an inhibition of redox signalling and an activation of PPARγ signalling. The ability of lycopene in inhibiting IL-8 production, NF-kB/p65 nuclear translocation, and redox signalling and in increasing PPARγ expression was also found in isolated rat alveolar macrophages exposed to CSE. These findings provide novel data on new molecular mechanisms by which lycopene regulates cigarette smoke-driven inflammation in human macrophages.

## Introduction

 Chronic obstructive pulmonary disease (COPD) is a syndrome characterized by progressive airflow limitation caused by chronic inflammation of the airways and lung parenchyma, which is due predominantly to chronic cigarette smoking [1]. Chronic exposure to cigarette smoke activates an inflammatory cascade in the airways resulting in the production of a number of cytokines and chemokines, with accompanying damage to the lung epithelium and increased vascular permeability and recruitment of macrophages and neutrophils [2], [3]. Macrophages are the major defence cells in the lower airways of the lung in healthy nonsmokers and appear to have an essential role in the pathogenesis of COPD by accounting for most known features of the disease [4]. Bronchoalveolar lavage (BAL) fluid from smokers compared to nonsmokers show a five-fold increase in the number of inflammatory cells in the lung, of which 85–90% are alveolar macrophages. Macrophages are predominant cells in the respiratory bronchioles of smokers; studies have shown a correlation between alveolar macrophage numbers and the extent of lung destruction in emphysema [5], [6].

The human chemokine IL-8 in particular, a member of the CXC chemokine family, activates adhesion molecules expression on endothelial cells [7] and it is an important activator and chemo-attractant for neutrophils [8] as well as T cells [9] and monocytes [10]. Increased levels of IL-8 have been found in induced sputum [11] and bronchoalveolar lavage from patients with smoking-related COPD associated with increased numbers of activated neutrophils [12] . Therefore, IL-8 has been implicated in the initiation and maintenance of chronic airway inflammation induced by cigarette smoke.

 Cigarette smoke harbors a multitude of chemical compounds, including high concentrations of free radicals and other oxidant species [13] and causes direct oxidative lung damage and indirect damage through the activation of various lung cells including alveolar macrophages [14]. Therefore, reactive oxygen species (ROS) present in smoke and phagocyte-derived ROS are intimately involved in the pathogenesis of smoking-related inflammation.

Nuclear factor-kB (NF-kB) is one of the redox-sensitive transcription factors involved in the inflammatory responses to cigarette smoke in the lungs and its activity is regulated by cytoplasmic degradation of the IkB inhibitor [15]. NF-kB dimers localize to the nucleus, once IkBα is inactivated, and undergo further modification, mostly through phosphorylation of the Rel proteins [15]. In the nucleus activated NF-kB binds to promoters of its target genes and regulates the expression of genes involved in many cellular events, including inflammation [16] through the activation of the Akt/phosphoinositide 3-kinase (PI3K) and the mitogen-activated protein kinase (MAPK) cascade [17]–[20].

It is known that peroxisome proliferator activated receptor-γ (PPARγ), a member of the ligand activated nuclear receptor superfamily, is able to regulate anti-inflammatory responses in cells exposed to cigarette smoke and that ligand-activated PPARγ is able to down-regulate NF-kB transcription. Recently, reports show that upregulation of phosphatase and tensin homolog deleted on chromosome 10 (PTEN), with the concomitant downregulation of PI3K-dependent signaling pathways [21]–[23], might be one of the mechanisms through which PPARγ agonists exert their anti-inflammatory actions.

Beneficial effects of tomato lycopene on the risk of smoke-related pathologies, including cancer and cardiovascular injury, have been found in epidemiological studies [24]. However, the experimental basis for such health benefits is not fully understood. One of the possible mechanisms for the protective activities of lycopene in smoke-related pathologies is by down-regulation of the cigarette smoke-stimulated inflammatory response [25], [26]. In fact, the carotenoid has been reported to inhibit pivotal pro-inflammatory mediators, including ROS [27] and cytokines [28] and to affect signal transduction pathways involved in inflammatory processes, including nicotinamide adenine dinucleotide phosphate oxidase oxidase [NADP(H)-oxidase] [28], MAPK [29], Akt/PI3K [30] and transcription factors, such as activator protein-1 (AP-1) [31] and NF-kB [31]–[35] and PPARγ cascade [28]. We recently reported that lycopene may inhibit ROS production, NOX-4 expression and cytokine release in human macrophages exposed to oxysterols [28]. Moreover, in the same model, it may enhance PPARγ expression [28].

To better understanding the role of lycopene in inflammatory processes caused by cigarette smoke, we investigated the effect of lycopene in modifying molecular pathways involved in cigarette smoke extract (CSE)-induced IL-8 production in human macrophages. Use of CSE remains a good practical model to study changes in cellular responses induced by cigarette smoke, since it mimics the *in vivo* soluble cigarette smoke components that are present during cigarette smoking. Here, we provide evidence of the inter-relationships between the signalling networks activated by cigarette smoke-induced stress and the anti-inflammatory effect of lycopene in macrophages.

## Results

### Lycopene inhibition of CSE-induced IL-8 production and NF-kB activation

Cigarette smoke induces a multitude of direct and indirect effects on lung tissue, but it is principally responsible for inflammation resulting in accumulation of macrophages and release of chemical mediators, which changes lung functions, morphology and gene expression. Since it has been reported that exposure to cigarette of macrophages stimulates release of different pro-inflammatory cytokines, including IL-8 [36] we measured the effect of different concentrations of CSE on intracellular IL-8 production in THP-1 cells incubated for 6 h and 24 h (Fig. 1A). CSE induced a dose- and a time- dependent increase in IL-8 production. A 6-h pre-treatment with lycopene at 2 µM, the maximum concentration which can be achievable in vivo after supplementation [37], down-regulated the production of IL-8 induced by CSE (Fig. 1B). Such an effect was dependent on the dose of carotenoid (Fig. 1C) and also occurred at mRNA levels (Fig. 1D). Similar results were found in the culture medium (Fig. 1E). A 6-h pre-treatment with lycopene reduced the increase of IL-8 production in culture medium induced by a 24-h treatment with CSE. These data show an anti-inflammatory potential of lycopene in CSE-exposed macrophages.

**Figure 1:** Effects of Cigarette smoke extract (CSE), alone and in combination with lycopene, on IL-8 production in human THP-1 cells. Panels A-D: intracellular IL-8 production; panel E: IL-8 production in culture medium. Panel A: effects of different CSE concentrations for 6 h and 24 h; panels B, D, E: effects of a pre-treatment for 6 h with lycopene (2 µM) followed by a 24-h CSE (0.5%) exposure; panel C: effects of a pre-treatment with different concentrations of lycopene followed by a 24-h CSE (0.5%) exposure; Panels A, B, C: representative Western Blot analyses; the values indicated represented the ratio of IL-8 and actin. Panel D: mRNA levels by reverse transcription polymerase chain reaction. Panel E: the values were the means ± SEM of three independent experiments. Panel E: the values were the means ± SEM of three independent experiments. Values not sharing the same letter were significantly different (P<0.05, Fisher's test).

Since it has been reported that IL-8 levels are modulated by NF-kB, we, then, investigated the effect of the specific NF-kB inhibitor pyrrolidine dithiocarbamate (PDTC) on CSE-induced IL-8 production in THP-1 cells. The pre-incubation of THP-1 cells with PDTC (10 µM) for 30 min prevented IL-8 protein production (Fig. 2A), demonstrating the key role of this transcription factor in CSE-stimulated IL-8 production by human macrophages. We further analysed the effects of CSE, alone and in combination with lycopene, on NF-kB DNA-binding activity in THP-1 cells. Nuclear extracts were prepared and NF-kB DNA binding activity was examined by EMSA. As shown in Figure 2B, a 3 h-treatment of the THP-1 cells with CSE resulted in an increase of the NF-kB DNA-binding activity. A 6-h pre-treatment with lycopene, at the concentration of 2 µM, inhibited CSE-mediated NF-kB DNA-binding activity. On the other hand, when compared to vehicle-control treated cells, no significant alterations in the DNA-binding activity were observed in lycopene alone-treated cells, suggesting that the NF-kB DNA-binding activity expression may not be substantially affected by physiological concentrations of the carotenoid. Moreover, CSE induced the translocation of NF-kB/p65 to the nucleus and lycopene pre-treatment suppressed it (Figure 2C). To determine whether the inhibitory action of lycopene towards NF-kB activation was due to its effect on IkBα degradation, the cytosolic levels of IKKα and IkBα were determined by Western blot analysis in cells treated with lycopene and CSE (Fig. 2D). Western blot analysis showed that CSE exposure resulted in phosphorylation of IKKα and pre-treatment of THP-1 cells with lycopene inhibited this phosphorylation (Fig. 2D). Further examining the effect of lycopene on IkBα phosphorylation by Western blot analysis, using an antibody that detects only the serine-phosphorylated form of IkBα, we found that CSE exposure resulted in increased phosphorylation of IkBα (Fig. 2D). Our data show that lycopene treatment of THP-1 cells suppressed this phosphorylation. These findings indicate that lycopene treatment of THP-1 cells resulted in inhibition of CSE-induced activation of IKKα, phosphorylation and degradation of IkBα, and subsequent activation of NF-kB.

**Figure 2:** Effects of lycopene on CSE-stimulated NF-kB activation in human THP-1 cells. Panel A: IL-8 production in culture medium after addition of the NF-kB inhibitor pyrrolidine dithiocarbamate (PDTC). THP-1 cells were pre-incubated with PDTC (10 µM) for 30 min and, then treated with CSE was added for 3 h and 24 h. Panel B: NF-kB DNA binding activity in cells pre-treated for 6 h with lycopene (2 µM) and, then exposed to CSE (0.5%) for 3 h; the specifity was demonstrated by using excess unlabeled NF-kB oligonucleotides ( = cold ssNF-kB) which competed away binding. Panel C: representative western blot analysis of nuclear NF-kB (p65)-associated proteins in cells pre-treated for 6 h with lycopene (2 µM) and, then exposed to CSE (0.5%) for 3 h; panel D: representative western blot analyses of cytosolic p-IKKα and p-IkBα in cells pre-treated for 6 h with lycopene (2 µM) and, then exposed to CSE (0.5%) for 3 h; the values indicated represented the ratio protein/actin. In panel A, values were the means ± SEM of three experiments. Values not sharing the same letter were significantly different (P<0.05, Fisher's test).

### Lycopene inhibition of CSE-stimulated redox signalling

It is known that NF-kB is activated by ROS and several lines of evidence suggest that cigarette smoke is a source of ROS. Moreover, cigarette smoke constituents can directly activate vascular ROS production through induction of NAD(P)H oxidase. Therefore, we measured ROS levels in the absence and in the presence of diphenyleneiodonium (DPI), an inhibitor of cellular NADPH oxidase in THP-1 cells exposed to CSE (Fig. 3A). Exposure of THP-1 cells to CSE, caused an increase in ROS production. Such an effect was evident at 3 h, and persisted at 24 h. When cells were pre-incubated with DPI at the concentration of 10 µM for 1 h and then washed prior to the addition of CSE, CSE-induced ROS production was abolished, suggesting that, at least in our experimental conditions, ROS production was generated intracellularly and not extracellularly by smoke. Pre-treatment of THP-1 cells with lycopene, at the concentration of 2 µM was able to prevent CSE-induced ROS production (Fig. 3B). Only slight and not significant inhibitory effects on ROS production by lycopene were observed in CSE-untreated THP-1 cells. The carotenoid was also able to inhibit the increase in NAD(P)H oxidase-4 (NOX-4) expression caused by CSE (Fig. 3C). Such an effect was evident at 3 h as well as at 24 h. Generation of oxidants by cigarette smoke appears to be the primary stimulus for activation of MAPK cascades. Whether the inhibitory effect of lycopene on CSE-induced ROS production extends to MAPK signalling pathway was investigated in THP-1 cells. Employing Western blot analysis, we found that a 3 h-CSE exposure resulted in a significant increase in the phosphorylation of JNK (Fig. 4A) ERK1/2 (Fig. 4B) and p38 (Fig. 4C) MAPK proteins in THP-1 cells. The levels of p-ERK1/2 were markedly higher than those of p-p38 and p-JNK. Pre-treatment with lycopene, at the concentration of 2 µM, resulted in a marked reduction in the CSE-induced phosphorylation of p38, ERK1/2 and JNK1/2 MAPK proteins, suggesting that the carotenoid is an effective inhibitor of these pathways.

**Figure 3:** Effects of lycopene on CSE-induced reactive oxygen species (ROS) production in human THP-1 cells. Panel A: ROS levels after addition of the NAD(P)H oxidase-4 (NOX-4) inhibitor diphenyleneiodonium (DPI) in cells exposed to CSE for 3 h and 24 h. Cells were pre-incubated with DPI at the concentration of 10 µM for 1 h and then washed prior to the addition of CSE. Panel B: ROS levels in cells pre-treated for 6 h with lycopene (2 µM) and, then exposed to CSE (0.5%) for 3 h and 24 h. Panel C: representative western blot analysis of NOX-4 in cells pre-treated for 6 h with lycopene (2 µM) and, then exposed to CSE (0.5%) for 3 h and 24 h; the values indicated represented the ratio NOX-4/actin. In panels A and B, values were the means ± SEM of five experiments. Values not sharing the same letter were significantly different (P<0.005, Tukey's test).

**Figure 4:** Effects of lycopene on CSE-induced MAPK phosphorylation in human THP-1 cells. Representative western blot analyses of JNK, ERK1/2 and p38 in cells pre-treated for 6 h with lycopene (2 µM) and, then exposed to CSE (0.5%) for 3 h. The values indicated represented the ratio phosphorylated protein/total protein.

### Lycopene enhancement of CSE-inhibited PPARγ signalling

PPARγ has been shown to regulate anti-inflammatory responses in CSE-exposed cells and ligand-activated PPARγ has been reported to down-regulate NF-kB transcription. Therefore, we measured the levels of PPARγ in THP-1 cells pre-treated for 6 h with lycopene and then exposed to CSE (Figs. 5A and 5B). Our results show that CSE decreased PPARγ at mRNA (Fig. 5A) and protein (Fig. 5B) levels. On the other hand, lycopene alone was able to increase the expression of this transcription factor at both mRNA and protein levels. Lycopene, in association with CSE, prevented the decrease in PPARγ levels induced by CSE, maintaining very high levels of this transcription factor.

**Figure 5:** Effects of lycopene on CSE-inhibited PPARγ signalling in human THP-1 cells. Panel A: PPARγ mRNA and panel B: representative western blot analysis of PPARγ protein cells pre-treated for 6 h with lycopene (2 µM) and, then exposed to CSE (0.5%) for 3 h. Panel C: representative western blot analysis of PTEN in cells pre-treated for 6 h with lycopene (2 µM) and/or with the PPARγ inhibitor GW9662 and, then exposed to CSE (0.5%) for 24 h. Panel D: representative western blot analysis of AKT in cells pre-treated for 6 h with lycopene (2 µM) and/or with the PPARγ inhibitor GW9662 and, then exposed to CSE (0.5%) for 24 h. GW9662 was pre-incubated at the concentration of 10 µM. The values indicated represented the ratio protein/actin (PTEN) and phosphorylated protein/total protein (AKT). In panel A, values were the means ± SEM of three experiments. Values not sharing the same letter were significantly different (P<0.05, Fisher's test).

Since PPARγ could exert its anti-inflammatory actions through an up-regulation of phosphatase and tensin homolog deleted on chromosome 10 (PTEN), THP-1 cells were treated with lycopene and CSE, alone and in combination, and PTEN expression was measured in the absence and in the presence of GW9662, an irreversible antagonist of PPARγ (Fig. 5C). Lycopene alone induced a ten-fold up-regulation of PTEN in THP-1 cells (Fig. 5C). Lycopene also induced an increase in the levels of PTEN in the presence of CSE (from 0.2 to 0.9), but this increase was much lower than that observed in cells treated with lycopene alone (0.9 *vs* 3.2), although PPARγ expression was not significant different in the two treatments. In contrast, CSE alone did not significantly modify PTEN expression, suggesting that the pro-inflammatory effects of CSE did not involve changes in this phosphatase. (Fig. 5C). However, the strong dependency of PTEN expression by PPARγ in cells treated with lycopene alone is suggested by the results obtained in the presence of GW9662. A 6-h pre-incubation with 10 µM GW9662 completely prevented the increase in PTEN expression induced by the carotenoid. GW9662 was also able to prevent the increase in PTEN expression induced by lycopene and CSE in combination, although in a minor extent.

It has been hypothesized that the up-regulation of PTEN could result in AKT inactivation. Therefore, we measured the levels of pAKT in THP-1 cells treated with lycopene and CSE, alone and in combination, in the absence and in the presence of GW9662 (Fig. 5D). Pre-treatment of THP-1 cells with lycopene induced a marked reduction in the CSE-induced phosphorylation of AKT, which was prevented by a 6-h pre-incubation with 10 µM GW9662 (Fig. 5D). These data suggest that the anti-inflammatory effects of lycopene (increase of PTEN expression and decrease in AKT phosphorylation) are PPARγ dependent. In contrast, THP-1 cells treated with CSE alone strongly increased AKT phosphorylation, but such an increase was independent of PPARγ, since pAKT expression was not modified by GW9662.

### Effects of lycopene on IL-8 expression, NF-kB/p65 nuclear translocation, ROS production and and PPARγ expression in isolated rat alveolar macrophages exposed to CSE

The ability of lycopene to modulate IL-8 production, redox and PPARγ signalling induced by CSE was also studied in rat alveolar macrophages (AMs) isolated from bronchoalveolar lavages (BALs). After the isolation of the cells and their incubation in culture conditions, the AMs were treated with lycopene and CSE, alone and in combination, in the experimental conditions indicated for THP-1 cells (Fig. 6). A 6-h pre-treatment with lycopene at the concentration of 2 µM was able to decrease CSE-induced IL-8 mRNA expression (Fig. 6A), NF-kB/p65 nuclear translocation (Fig. 6B), ROS production (Fig. 6C) and to increase PPARγ expression (Fig. 6D), confirming a key role of lycopene in the inhibition of inflammatory response induced by cigarette smoke.

**Figure 6:** Effects of lycopene, alone and in combination with cigarette smoke extract (CSE), on intracellular IL-8 mRNA levels, NF-kB/p65 nuclear translocation, ROS production and PPARγ expression in isolated rat alveolar macrophages (AMs). Panel A: IL-8 levels by reverse transcription polymerase chain reaction in cells treated for 6 h with lycopene (2 µM) followed by a 24-h CSE (0.5%) exposure. Panel B: representative western blot analysis of nuclear NF-kB (p65)-associated proteins in cells pre-treated for 6 h with lycopene (2 µM) and, then exposed to CSE (0.5%) for 3 h. Panel C: ROS levels in cells pre-treated for 6 h with lycopene (2 µM) and, then exposed to CSE (0.5%) for 3 h. Panel D: PPARγ: representative western blot analysis of PPARγ protein in cells pre-treated for 6 h with lycopene (2 µM) and, then exposed to CSE (0.5%) for 3 h. In panels A and C, values were the means ± SEM of three experiments. Values not sharing the same letter were significantly different (P<0.05, Fisher's test).

## Discussion

It is widely recognized that cigarette smoke caused an inflammatory response [1]. According with this, smoking is the major risk factor for chronic obstructive pulmonary disease (COPD) and lung fibrosis, pathological processes characterized by pulmonary leukocyte infiltration, chronic inflammation and progressive tissue destruction [1]. It has been reported that exposure to cigarette smoke of cultured human blood monocytes or macrophagic cultures stimulates release of several pro-inflammatory cytokines, including IL-8 [38]–[45]. In addition, fibroblasts [46]–[48] bronchial [49], [50] and alveolar [51] epithelial cells, which are the primary target for any inhaled environmental agent, have been reported to release IL-8, when exposed to cigarette smoke. In our study, the acute exposition to CSE up-regulated IL-8 expression of human THP-1 macrophages at both mRNA and protein levels in a dose- and a time-dependent manner. In contrast, pre-treatment with lycopene, in a range of concentrations which can be achievable *in vivo* after supplementation [37], was able to counteract this effect, suggesting that the carotenoid may have a key role in regulating smoke-induced inflammatory processes. This finding is in agreement with previous observations showing a down-regulation of pro-inflammatory cytokine expression by lycopene in *in vitro* and *in vivo* models [28], [52]–[56]. An inhibition of pro-inflammatory cytokine levels, including IL-8, has been observed following treatment with other carotenoids, including β-carotene [57], [58]. In particular, β-carotene has been reported to arrest the increase in IL-6 and IL-8 induced by a long-term cigarette smoke exposition in serum, bronchoalveolar lavage fluid and lung tissue of rats [57]. Moreover, β-carotene had an inhibitory effect on IL-8 and TNF-α secretion in phorbol-12-myristate-13-acetate-stimulated HL-60 cells, although such an inhibition was observed at low (2 µM) but not at high (20 µM) carotenoid concentrations [58]. In agreement with the literature [49], [59]–[61] our data show that the production of the pro-inflammatory cytokine IL-8 by CSE is strongly linked to activation of NF-kB, since PDTC, a chemical that stabilizes the NF-kB/IkB-α complex [62] and inhibits the nuclear translocation of activated NF-kB, significantly inhibited it. Therefore, lycopene potential ability to influence cytokine levels may be, at least in part, explained by carotenoid localization in or within cell membrane, modulating surface molecules for primary immune response, which activate signalling pathways responsible for modulation of NF-kB. According with this hypothesis, our data also show that lycopene may counteract the effect of CSE on NF-kB activation. The inhibition of NF-κB DNA binding activity by lycopene was mediated through the downregulation of IKKα and IκB phosphorylation, and NF–κB p65 subunit translocation from cytosol to nucleus. Increasing evidence suggests that lycopene inhibited the binding activity of NF-κB [32], [33]. Moreover, tomato lycopene extract prevented lipopolysaccharide (LPS)-induced pro-inflammatory gene expression by blocking NF-kB signalling [35]. Based on data showing that one of the early events occurring in smoke-exposed cells is the increase in ROS levels, we examined the possibility that ROS were involved in NF-kB activation. We believe that the intracellularly generated ROS trigger the effects of smoke in THP-1 cells, on the basis of our experiments showing that diphenyleneiodonium (DPI), an inhibitor of cellular NADPH oxidase, was able to abolish the presence of ROS in CSE-exposed macrophages. Concomitantly, CSE was able to increase NOX-4 expression in THP-1 cells. In our study, lycopene inhibited both CSE-induced ROS production and CSE-stimulated NOX-4 expression. This is not surprising since the carotenoid has been reported to act as an intracellular redox agent, at least *in vitro* conditions [26]. Due to its extended system of conjugated double bonds, lycopene can effectively quench singlet oxygen [27] and free radicals [63] generated by smoking exposure. Moreover, recent data suggest that the carotenoid may also inhibit NOX-4 expression in human macrophages exposed to oxidants [28], [64].

The MAP kinases (ERK1/2, p38 and JNK) have been reported to be activated by oxidant stimuli and to mediate production of cytokines via NF-kB activation [25], [65]–[67]. Whether the inhibitory effect of lycopene on CSE-induced NF-kB activation pathway extends to MAPK signalling pathway was investigated. Employing Western blot analysis, we found that CSE exposure to THP-1 cells resulted in a significant increase in the phosphorylation of p38, ERK1/2, and JNK1/2 MAPK proteins. On the other hand, lycopene treatment resulted in a marked reduction in the CSE-induced phosphorylation of the three redox-sensitive MAPK proteins as shown in Figure 4, suggesting that lycopene is an effective inhibitor of MAPK pathways in THP-1 cells. The findings that lycopene can reduce MAPK activation in human macrophages confirm previous evidence in LPS-stimulated murine bone marrow-dendritic cells [29] and in oxysterol-exposed THP-1 cells [28] .

It has been reported that nicotine and the tobacco-specific carcinogen 4-(methylnitrosamino)-1-(3-pyridyl)-1-butanone, two components of cigarette smoke, induce phosphorylation of AKT (pAKT) in non-immortalized human airway epithelial cells [68]. Moreover, pAKT has been reported to activate NF-kB signalling and the consequent expression of pro-inflammatory cytokines. We therefore tested the effect of lycopene on CSE-induced activation of AKT. For this, protein lysates were analysed by Western blot using antibodies that detect the phosphorylated form of this protein. As shown in Figure 4, CSE exposure to THP-1 cells resulted in increased AKT phosphorylation, and lycopene treatment suppressed it.

A recent *in vitro* study also suggests that lycopene may have a key role in the modulation of AKT pathway under smoke conditions [30]. In fact, while RAT-1 fibroblasts exposed to cigarette smoke condensate exhibited high levels of phosphorylated AKT, cells exposed to a combination of tar and lycopene strongly decreased them. Moreover, in the same study, the expression of the heat shock protein (hsp)90 was increased following tar exposure [30]. Such an increase was counteracted by lycopene. This finding is particularly interesting in view of a previous report showing that hsp90 maintains Akt activity by binding to Akt and by preventing PP2A-dependent dephosphorylation of Akt [69]. Moreover, hsp90 has been reported to prevent proteasome-dependent degradation of PDK1, which is known to activate Akt.

PPARγ has been implicated in anti-inflammatory response and increasing evidence suggests that cigarette smoke strongly reduced it [70]. PPARγ activation has been shown to inhibit pro-inflammatory cytokine production by preventing activation and translocation of NF-kB [71]. In our study, lycopene was able to increase PPARγ at both mRNA and protein levels, confirming previous reports [28]. Moreover, the carotenoid, counteracted the decrease in PPARγ induced by CSE. Recently, it has been shown that upregulation of phosphatase and tensin homolog deleted on chromosome 10 (PTEN), with the concomitant downregulation of PI3K-dependent signaling pathways, might be another mechanism through which PPARγ exerted its anti-inflammatory actions. Therefore, we investigated the effects of lycopene on PTEN expression. Pre-treatment of THP-1 cells with the carotenoid increased PTEN expression and decreased Akt phosphorylation. However, it should be pointed out that the increase in PTEN expression by lycopene in the presence of CSE was much lower than that observed in the presence of lycopene alone, although PPARγ expression was not significant different in the two treatments. Interestingly, GW9662, which is an irreversible antagonist of PPARγ, prevented the increase in PTEN and the decrease in pAKT induced by lycopene, suggesting that PTEN activation required an increase in PPARγ levels and antagonized the phosphorylation of Akt. It has been suggested that lycopene may have a PPARγ agonist activity [72], [73]. In THP-1 cells [72] as well as in LNCaP cells [73], the specific antagonist of PPARγ (GW9662) reverted the PPARγ-mediated effects of lycopene on cholesterol metabolism [72] and/or cell proliferation [72], [73]. In addition, Sharoni and colleagues have proposed that some carotenoids, such as lycopene, phytoene, phytofluene, and β-carotene cause the transactivation of peroxisome proliferator response element in cells co-transfected with PPARγ [74]. In contrast, CSE alone did not exert pro-inflammatory effects through a down-regulation of PPARγ expression, since CSE treatment did not significantly affect PTEN expression and the increase in CSE-induced AKT phosphorylation was unaffected by GW9662.

In conclusion, CSE exposure of human THP-1 macrophages caused an increase in the levels of the pro-inflammatory cytokine IL-8 which occurred through activation of NF-kB. Pre-treatment of cells with lycopene decreased both CSE-induced IL-8 production and NF-kB activation. Two mechanisms, could be implicated in such anti-inflammatory response of lycopene. The first one involves an interference with redox signalling, demonstrated by decrease in ROS production and in redox-sensitive MAPK activation by lycopene. The second one involves, at least in part, a PPARγ-dependent activation of PTEN which results in Akt inactivation. These findings thus represent a direct evidence that lycopene may act as an anti-inflammatory compound in cells exposed to cigarette smoke and provide novel data on important molecular mechanisms by which lycopene regulates cigarette smoke-driven NF-kB-dependent inflammation in human macrophages.

## Materials and Methods

### Cell culture

THP-1 (American Type Culture Collection, Rockville, MD, USA) were grown in RPMI Dutch Modified (Sigma, Milan, Italy) without antibiotics and supplemented with 10% fetal calf serum, non essential aminoacids, 2 mM glutamine, and 1 mM sodium piruvate**.** Cells were maintained in log phase by seeding twice a week at density of 3×10^8^ cells/L at 37°C under 5% CO_2_/air atmosphere. Lycopene (LycoRed Natural Products Industries Ltd, Beer Sheva, Israel) was delivered to the cells (10^9^ cells/L) using tetrahydrofuran (THF) as a solvent. To avoid the formation of peroxides, the solvent contained 0.025% butylated hydroxytoluene (BHT). The stock solutions of lycopene were prepared immediately before each experiment. From the stock solutions, aliquots of lycopene were rapidly added to the culture medium to give the final concentrations indicated. Control cultures were treated with THF + BHT. The amount of THF added to the cells was not greater than 0.5% (v/v) and it was the same in control cells as well as in treated ones. No differences were found between cells treated with THF and untreated cells in terms of cell viability and ROS production. After the addition of lycopene for 6 h, the medium was not further replaced throughout the experiments. Experiments were routinely carried out on triplicate cultures. At the times indicated, cells were harvested and quadruplicate haemocytometer counts were performed. The trypan blue dye exclusion method was used to evaluate the percentage of viable cells. No differences were found between vehicle control- and lycopene-treated cells, in the range of carotenoid concentration indicated, in terms of cell viability.

### Isolation and culture of rat alveolar macrophages AMs

Male Wistar rats (232–305 g body weight) (Catholic University laboratories, Rome, Italy) were used for isolation of AMs. After rats were anesthetized by an intraperitoneal injection of ketamine (90 mg/kg) and xylazine (5 mg/kg), the trachea were cannulated and AMs were obtained by three bronchoalveolar lavages (BALs) using 10 ml of Ca2+− and Mg2+−free DPBS each time. Cells recovered from the pooled BAL fluid were suspended in MEM containing 0.02% BSA, 25 mM HEPES, 100 U/ml of penicillin, and 100 µg/ml of streptomycin. The cells were seeded in either 24-well culture plates or 35 mm-diameter culture dishes. After incubation for 2 h at 37°C in a 5% CO_2_ humidified atmosphere to allow AMs to adhere, non-adherent cells were removed by washing one time with complete medium. AMs were incubated overnight to make them quiescent. Cell viability as determined by trypan blue exclusion was >95% and the purity of AMs as determined by non-specific esterase staining (Sigma- Aldrich) was >90%. AMs from the same rat were used for the same series of experiments to reduce inter-individual variation. All animal procedures were reviewed and approved by the Ministry of Health, Veterinary Service, Rome, Italy.

### Preparation of aqueous cigarette smoke extract

Research grade cigarettes (1R3F) were obtained from the Kentucky Tobacco Research and Development Center at the University of Kentucky (Lexington, KY). The total particulate matter (TPM) content of 1R3F was 17.1 mg/cigarette, tar (15 mg/cigarette) and nicotine (1.16 mg/cigarette). A 10% cigarette smoke extract (CSE) was prepared by bubbling smoke from one cigarette into 10 ml of culture medium supplemented with 1% FBS at a rate of one cigarette per minute as described previously, using a modification of the method described by Carp and Janoff [75]. The pH of the CSE was adjusted to 7.4 and was sterile filtered through a 0.45-µm filter (25-mm Acrodisc; Pall, Ann Arbor, MI). The CSE preparation was standardized by monitoring the absorbance at 320 nm (optical density of 0.74±0.05). The spectral variations observed between different CSE preparations at 320-nm wavelength were found to be within the acceptable limits. CSE was freshly prepared for each experiment and diluted with culture medium containing 1% FBS immediately before use. Control medium was prepared by bubbling air through 10 ml of culture medium supplemented with 1% FBS, adjusting pH to 7.4, and sterile filtered as described for 10% CSE. The final concentration of CSE was 0.5%. At this concentration, cell viability was always greater than 95% as measured by trypan blue exclusion.

### Chemiluminescence Immunometric Assay of IL-8

IL-8 was measured by a solid-phase, two-site chemiluminescence immunometric assay (Siemens Medical Solution Diagnostics, LA, CA, USA). The intra and inter-assay CV for IL-8 was <3.8 % and 6.7%. The detection limit was 2.0 pg/ml for IL-8.

### Measurement of ROS

Cells were harvested to evaluate reactive oxygen species (ROS) production using the di(acetoxymethyl ester) analog (C-2938) of 6-carboxy-2′,7′-dichlorodihydrofluorescein diacetate (DCF) (Molecular Probes, Inc., Eugene, OR) as described [76]. Before the addition of the fluorescent probes, 2×10^6^ cells were washed to eliminate the amount of lycopene not cell-associated. Fluorescent units were measured in each well after 30 min incubation with DCF (10 µM) by use of a Cytofluor 2300/2350 Fluorescence Measurement System (Millipore Corp., Bedford, MA). Lycopene did not alter the basal fluorescence of DCF.

### Preparation of whole cell lysates, cytosolic and nuclear extracts

Cells (10×10^6^) were harvested, washed once with ice-cold phosphate-buffered saline (PBS), and gently lysed for 30 min in ice-cold lysis buffer (1 mM MgCl2, 350 mM NaCl, 20 mM N-2-hydroxyethylpiperazine-N′-2-ethane sulfonic acid (HEPES), 0.5 mM ethylenediaminetetraacetate (EDTA), 0.1 mM ethyleneglycol-bis(β-aminoethyl ether)-N,N′-tetraacetic acid (EGTA), 1 mM dithiothreitol (DTT), 1 mM Na4P2O7, 1 mM PMSF, 1 mM aprotinin, 1.5 mM leupeptin, 1 mM Na_3_VO_4_, 20% glycerol, 1% NP40). Cell lysates were centrifuged for 10 min at 4°C (10,000 g) to obtain the supernatants (whole cell lysate). For the cytosolic extracts, the confluent cells were washed in ice-cold PBS, suspended in ice-cold hypotonic buffer (10 mM HEPES, pH 7.9), 1.5 mM MgCl2, 10 mM KCl, 0.3% NP-40, 0.1 mM EDTA, 0.1 mM EGTA, 0.5 mM DTT, 0.1 mM PMSF, 0.1% aprotinin), and lysed for 15 min on ice. The lysates were centrifuged for 10 min at 10 000×g. The supernatants were designated as cytosolic extracts. The nuclear pellet was resuspended in the high salt lysis buffer (10 mM HEPES, 1.5 mM MgCl2, 420 mM NaCl, 0.2 mM EDTA, 0.1 mM EGTA, 25% glycerol, 0.5 mM DTT, 0.1 mM PMSF, 0.1% aprotinin), and incubated at 4°C for 30 min. The resulting supernatants were reserved as nuclear extracts. The protein concentrations of samples were determined by Bio-Rad (Hercules, CA, USA) protein assay.

### Western blot analysis of IL-8, p65, p-IKKα, p-IkBα, IkBα, Nox-4, p38 and p-p38, ERK1/2, pERK1/2, JNK, p-JNK, PPARγ, AKT, p-AKT and PTEN expression

The anti-IL-8 (H-60, Cat. no. SC-7922), anti-NOX-4 (N-15, Cat. No. sc-21860), anti-p38 (C-20, Cat. No. SC-535), anti-ERK1/2 (K-23, Cat. No. SC-94), , anti-JNK (C-17, Cat. No. SC-474), , anti-PPARγ (H-100, catalog. no. SC-7196), anti-AKT (C-20, Cat. no. SC-1618), anti-pAKT (anti-p-Akt1/2/3 (Thr 308-R, catalog. no. sc-16646-R), and anti-IKK (M280, Cat. no. SC-7182) polyclonal antibodies and the anti-p65 (F-6, Cat. No. SC-8008), p-p38 (D-8, Cat. No. SC-7973), anti p-ERK1/2 (E-4, Cat. No. SC-7383), anti-p-JNK (G-7, Cat. No. SC-6254) and anti-PTEN (28H6 , Cat. No. SC-56205) monoclonal antibodies were purchased from Santa Cruz Biotechnology (Santa Cruz, CA). The anti- IkBα and the anti-p-IkBα (Ser32/36) monoclonal antibodies were obtained from Cell Signaling Technology (Beverly, MA, USA). The blots were washed and exposed to horseradish peroxidase-labeled secondary antibodies (Amersham Pharmacia Biotech, Arlington Heights, IL) for 45 min at room temperature. The immunocomplexes were visualized by the enhanced chemiluminescence detection system and quantified by densitometric scanning.

### RT-PCR of IL-8 and PPARγ

Total RNA was extracted from cells samples using Trizol according to manufacturer's protocols (Invitrogen life technologies, Paisley U.K.) the RNA was eluted in DEPC treated water (0.01% DEPC) and stored at −80° until RT-PCR analysis. Nucleic acid concentrations were measured by spectrophotometry (Hewlett-Packard HP UV/VIS spectrophotometer 8450).

RT-PCR assay was performed using the two-step method. For the first-step of reverse transcription, we used QuantiTect Reverse® Trancription kit (Qiagen, Hilden, Germany) with 500 ηg of total RNA as template RNA, following the manufacturer's procedure. For the second step of real time PCR reactions, we employed QuantiTect SYBR® Green Kits (Qiagen) and QuantiTect® Primer Assays (Qiagen) for human and rat β-Actin, IL-8, PPARγ, according to manufacturer's protocol described for the real-time thermalcycler LightCycler (Roche). PCR data obtained by the LightCycler software were automatically analysed by the Relative Quantification Software (Roche) and expressed as target/reference ratio. Our approach was based on the calibrator-normalized relative quantification including correction for PCR efficiency.

### Electrophoretic Mobility-Shift Assay

Frozen cell pellets were processed to obtain nuclear extracts. The pellet was treated as indicated in [35]. Binding reactions containing 5 µg nuclear extracts, 10 mmol/L Tris-HCl (pH 7.6), 5 % glycerol, 1 mmol/L EDTA, 1 mmol/L DTT , 50 mmol/L NaCl, and 3 mg poly(dI-dC) were incubated for 30 min with 5,000 cpm of α-^ 32^P-end-labeled double-stranded oligonucleotide in a total volume of 20 µL. The probe was 5′-AGTTGAGGGGACTTTCCCAGGC3′. Labeling of the probe was obtained by incubating 5 pmol of oligonucleotide with 10 pmol [α-^32^P]ATP and 3 UT4 polynucleotide kinase for 30 min at 37°C. The probe was then purified with MicroBIO-Spin P-30 columns. Complexes were separated on 60 g/L polyacrylamide gels with 45 mmol/L Tris-borate, 1 mmol/L EDTA, pH 8 buffer. After fixation and drying, gels were exposed on phosphor screens which were then analyzed by phosphor/fluorescence imager STORM 840 (Molecular and Dynamics, Sunnyvale, CA, USA). The intensity of the revealed bands was directly quantified by Image QuaNT software (Molecular Dynamics, Sunnyvale, CA, USA).

### Analysis of p65 protein

Nuclear extracts, 25–30 µg of protein, were separated by sodium dodecyl sulfate polyacrilamide gel electrophoresis with 40–120 g/L Bis-Tris gels (NOVEX, San Diego, CA, USA) and transferred to Immobilon-P membranes (Millipore Corp, Bedford, MA, USA) with the use of a semidry system. Immunoblots were blocked overnight at 4°C in 50 g/L dried milk in PBS, pH 7.4 plus 0.05% Tween 20. Blots were incubated with polyclonal primary antibodies to p65 (Santa Cruz, Biotechnology, CA, USA, clone 49.Ser 311, catalog no. SC-135769) in PBS plus 0.05% Tween 20 for 1–2 h at room temperature. The blots were visualized as described in Western blotting assay.

### Statistical analysis

Three separate cultures per treatment were utilized for analysis in each experiment. Values were presented as means ± SEM. One-way ANOVA was used to determine differences between the treatments in Figs. 1D, 1E, 2A, 5A, 6A, 6C. When significant values were found (P<0.05), post hoc comparisons of means were made using Fisher's test. Multifactorial two-way analysis of variance (ANOVA) was adopted to assess any differences among the treatments and the times in Figs. 3A, 3B. When significant values were found (P<0.05), *post hoc* comparisons of means were made using the Tukey's Honestly Significant Differences test. Differences were analyzed using Minitab Software (Minitab, Inc., State College, PA).
